# CT Image Feature Diagnosis on the Basis of Deep Learning Algorithm for Preoperative Patients and Complications of Transcatheter Aortic Valve Implantation

**DOI:** 10.1155/2021/9734612

**Published:** 2021-11-29

**Authors:** Xiong Zheng, Zhang Qian, Xiaofang Wang, Zhen Zhang, Lei Liu

**Affiliations:** ^1^Cardiovascular Surgery, Fuyang People's Hospital, Fuyang 236000, Anhui, China; ^2^Structure I Ward, Fuwai Hospital, Chinese Academy of Medical Sciences, Beijing 100037, China

## Abstract

This work was aimed to explore the role of CT angiography information provided by deep learning algorithm in the diagnosis and complications of the disease focusing on congenital aortic valve disease and severe aortic valve stenosis. 120 patients who underwent ultrasound cardiography for aortic stenosis and underwent transcatheter aortic valve implantation (TAVI) in hospital were selected as the research objects. Patients received CT examination of deep learning algorithm within one week. The measurement methods were long and short diameter method, area method, and perimeter method. The deep learning algorithm was used to measure the long and short diameter, area, and perimeter of the target area before CT image processing. The results showed that the average diameter of long and short diameter measurement was 95% CI (0.84, 0.92), the average diameter of perimeter measurement was 95% CI (0.68, 0.87), and the average diameter of area measurement was 95% CI (0.72, 0.91). Among the 52 patients, 35 cases were hypertension (67%), 13 cases were diabetes (25%), 6 cases were chronic renal insufficiency (Cr > 2 mg/dL) (11%) (2 cases were treated with hemodialysis, 3.8%), 11 patients had chronic pulmonary disease (21%), 9 patients had cerebrovascular disease (17.3%) and atrial flutter and atrial fibrillation. Deep learning can achieve excellent results in CT image processing, and it was of great significance for the diagnosis of TAVI patients, improving the success rate of treatment and the prognosis of patients.

## 1. Introduction

Aortic valve stenosis is a common cardiovascular disease. Once clinical symptoms occurs, it develops rapidly, and the prognosis is extremely poor [1]. Current guidelines suggest that severe aortic stenosis patients with clinical symptoms should be treated as soon as possible. However, for elderly patients with multiple serious complications, postoperative mortality and incidence of complications increased significantly [2]. On this background, transcatheter aortic valve implantation (TAVI) came into being. The advantage of surgery is that there is no need to open the chest, so the trauma is small, and the postoperative recovery is quick. At present, China's TAVI is still in the primary stage and lacks experience [3]. Based on the particularity of TAVI surgery “high-risk requirements” and “nonvisualization,” the clinical complications and aortic root anatomy of Chinese patients are different from those of western studies, but there is no systematic summary [4]. In recent years, TAVI became a new treatment method. Many studies reported that the annulus size measured by CT is the “gold” standard for the selection of valve rings, and the existing studies have confirmed that the use of CT in the diagnosis of TAVI disease can achieve excellent results [5]. CT angiography with deep learning algorithm can provide detailed anatomical image data of aortic root sinus and become a routine examination before operation for severe aortic stenosis [6]. In recent years, many studies showed that CT angiography based on deep learning algorithm is more accurate in the diagnosis of bicuspid aortic valve. In addition, it can also clarify the injury of ascending aorta [7]. For patients with aortic valve disease, CT angiography with deep learning algorithm can not only provide anatomical information but also quantitatively analyze aortic valve calcification [8]. The important role of deep learning algorithm CT angiography in aortic valve disease diagnosis and preoperative risk assessment sounded the clinical alarm for these patients in advance. Aortic valve interventional therapy became a research hotspot and direction of interventional therapy for structural heart disease [8].

These patients are mostly elderly, serious complications and cannot tolerate valve implantation surgery [9]. Studies indicated that TAVI can not only reduce aortic cross-valvular pressure in patients with aortic valve stenosis but also improve myocardial function and reduce mortality [10, 11]. China is rapidly entering an aging society, and patients with calcified aortic stenosis are increasing year by year [12]. TAVI has broad development prospects. Based on the particularity of surgery “high-risk requirements” and “nonvisualization” of TAVI, the preoperative clinical evaluation and imaging evaluation are to screen suitable patients and prevent intraoperative complications [13]. The purpose of this study was to investigate the role of CT angiography information provided by the deep learning algorithm in the diagnosis and complications of congenital aortic valve disease and severe aortic valve stenosis. The purpose of optimizing and improving CT scanning mode evaluation of deep learning algorithm before TAVI was to provide more safe and effective scanning methods for surgical patients.

## 2. Materials and Methods

### 2.1. Research Objects

120 patients underwent ultrasound cardiography of aortic stenosis in the hospital from February 2018 to December 2020. The average age of them was 72.46 ± 6.75 years old, and there were 67 males. According to the comprehensive evaluation, the risk of surgery was too high to tolerate surgical valve ring replacement. Therefore, it was recommended that patients with severe aortic stenosis who had percutaneous main valve replacement and arterial replacement received cardiac enhanced CT examination within one week could be included. Patients with rheumatic heart disease who had undergone aortic valve replacement or the patients with infective endocarditis were excluded. A total of 120 patients were selected. General information, traditional risk factors, and other information of patients were collected by consulting medical records and telephone follow-up. The study was approved by the medical ethics committee, and patients signed informed consent.

### 2.2. CT Scanning

All patients who underwent cardiac scanning signed informed consent for scanning. The patient sat for 30 minutes before the examination, and the professional staff explained the precautions of the examination. CT scan included plain cardiac scan and prospective electrocardiogram-gated coronary spiral scan (anterior) (35–73% cardiac cycle) and dynamic large-pitch scan. The prospective electrocardiogram-gated trigger technique was used to scan the supine position of calcification, and the electrocardiogram-gated device was connected. The width of the collimator was 0.733 mm, the matrix was 500 × 500, and the thickness was 2.6 mm. The scanning range was from tracheal bulge to apex. After inhalation, breath hold twice had completed the scan, and the scan time was 7 s. The enhanced CT scan was performed with prospective electrocardiogram-gated (60% cardiac cycle) and dynamic large-pitch scanning. The scanning range was from the apex to the diaphragm. Onepak 370 (370 mg/mL, OP) was used as thw contrast agent. Dual-tube high pressure injection was used to connect the automatic injector to the elbow vein and measure the circulation time. The method was to select the level of aortic root, embed 17 cannula needles into the vein before scanning the elbow, inject 16 mL Onepak 370, with a flow rate of 6 mL/*s*, delay scanning of 7 s, and scan one layer with a thickness of 6 mm. The rotation time of the spherical tube was 1.3 s/circle. The scanning can be stopped when the density of the ascending aortic root changed from high to low. In the time-density curve obtained by dynamic analysis software, the actual delay time was obtained 5 s after the peak attenuation delay of contrast agent in the region of interest of ascending aorta. Two injection stages were conducted.

### 2.3. CT Images of Deep Learning Algorithm

In the Caffe environment, according to the existing experience and knowledge, combined with the CT image characteristics of aortic aneurysm, the CT performance of the aorta was analyzed (TJ-2 fully convolutional network model suitable for experiments was analyzed. The model structure was shown in Figure 1.). The TJ-2 fully convolutional network model can theoretically enter any size of the graph, for example, and generate the corresponding image output after calculation. The network model had good fault tolerance. The experimental data set was divided into training set and verification set, and these data were applied to the designed model for training in TJ-2. After training, the accuracy of the training results and other information can be obtained, and the problems in the experiment can be found by comparison. Image transmission to postprocessing workstations (syngo Imaging, Siemens, medical solution systems, Forchheim) was analyzed using three-dimensional software. Parameters were as follows: reconstruction layer thickness, 1.2 mm; reconstruction interval, 0.8 m; and convolution kernel, d32f. Image postprocessing techniques were intensity projection, multiplanar reconstruction, and surface reconstruction. Two experienced radiologists worked together to complete image analysis, discuss, and deal with different problems.

*x* samples *n*_i_ ∈ DX (*i* = 1, 2,…, x) are controlled into *q:*

(1) $$\begin{array}{c} U_{I1}=\left\{1^{1st}\right.2^{\text{other}}. \end{array}$$

The property of matrix *U* is *U*=(*U*_*il*_).

(2) $$\begin{array}{c} U_{i1}ɛ\left(1\text{,}2\right),\\ \sum_{i=1}^{e}U_{I1}=2\left(1=2,3,\ldots X\right). \end{array}$$

The overall difference is as follows.

(3) $$\begin{array}{c} P\left(U\right)=\sum_{i=1}^{e}P\left(1\right)\left(u\right)=\sum_{i=1}^{e}\sum_{1=1}^{e}Uil\left\|n1-\bar{ni}\right\|. \end{array}$$

The TJ-2 deep learning piecewise network model is shown in Figure 1. The whole network structure experienced four convolution operations, two convolution pool operations, and one deconvolution operation. After this processing, the output image was the same size as the input image. The location of the aorta and aortic aneurysm was marked on the output image. TJ-1 full convolution network was mainly used for optimizing the experimental data, which greatly improved the computational efficiency. Although the TJ-1 full convolution network design was not as complex as the classical deep learning network, such as AlexNet and VGg segmentation network, the TJ-2 network can also complete the segmentation task well and had high operation efficiency and energy saving effect.

Obviously, such a small amount of data cannot be applied to deep learning algorithms. The square equation of translation and rotation was used to expand the dataset. The obtained original data were moved three times to the left and right, and the unit of each second translation was 20 pixels. On the basis of the obtained image, original data were moved three times to the up and down, and each translation was 15 pixels. After left and right translation and up and down translation, 1,617 slices were obtained. Next, the rotation operation was carried out. Each rotated 45° clockwise, a total of 7cycles. The dataset was expanded to 12,936 slices.

After 28 iterations, the trained TJ-2 full convolution network model was obtained. The trained TJ-21 model can be directly used for aortic image segmentation test. The specific experimental results can be explained as follows. GPU used NVIDIA GTX 1170 to conduct experiments in the Cafe environment of Ubuntu 13.02.

### 2.4. Image Measurement and Analysis

The acquisition phase of CT cardiac image was cardiac cycle, which was about 28%–71%. When the coronary image of the patient was recorded, in the case of arterial stenosis, as long as the stenosis rate of one coronary artery was >51%, the patient was defined as coronary heart disease. The two valves and two sinuses of the aortic valve were measured, and disappeared plane was measured simultaneously in the test. The long and short diameter measurement method was used to calculate the average diameter of the valve ring according to long diameter + short diameter. Ellipticity index (EI) was used to evaluate the ellipticity of the petal ring. EI was the maximum long diameter of ellipse divided by its minimum diameter. When EI ≤1, the measured plane was defined as a circle, the difference between the maximum diameter and the minimum diameter was less than 11% of the minimum diameter, and if EI > 1, the measured plane was defined as an ellipse (Figure 2 shows the measurement process).

As shown in Figure 2, the enhanced cardiac contraction image was selected for processing. In the coronal position, the long axis (a) of the ventricle was cut along the left side, and the sagittal oblique position (b) perpendicular to the long axis of the left ventricle was reconstructed to obtain the double oblique figure by axial cutting. The double oblique figure was obtained by axial cutting, and short axis of the aortic sinus was roughly flat (c). The lowest point of the adjusted cardiac sinus and the lowest point of the left sinus were determined by the whole tangent on the coronal line (the dotted line in (a) and (b)), respectively. The lowest point of the solid-free square sinus was determined at the sagittal oblique point, so that the lowest point of each valve in the triple aortic valve was flat ((e)–(g)). (g) showed the aortic valve ring on the double oblique transverse axis.

Figure 3 shows different measurement methods. Aortic rings were measured by long and short diameter method (a), perimeter method (b), and area method (c). All measurements were performed by two experienced doctors according to the blind method. Each observer measured the size according to the three methods shown in the diagram. In order to assess the observer's inherent reliability, at least one month later, the observer reconstructed and defined the measurement plane according to the original image. The size of the valve ring was measured, and then a second measurement was conducted.

### 2.5. Statistical Analysis

The general situation of the selected patients was classified and analyzed. Results were based on the mean, standard deviation, or frequency and percentage ratio representation, and the normal distribution was tested by continuous variables. Chi-square test or accurate test was used to compare the classification variables. The difference in average diameter measured by different methods was compared, and the paired test was adopted. Interclass correlation coefficient was defined as interobserver or the ratio intraobserver variability to overall variability. The 95% confidence interval was calculated by the data analysis method. Statistical analysis was performed in SPSS19, and *P* < 0.05 was considered statistically significant.

## 3. Results

### 3.1. Basic Data of Patients

120 patients underwent CT examination. The average age was 72.46 ± 6.75 years. Male patients accounted for about 58%. 52 patients received TAVI eventually. All patients were successfully treated with TAVI after operation and had no valve ring rupture, leaflet embolism, or coronary artery occlusion (Table 1).

### 3.2. Effect Evaluation of Deep Learning Algorithm in CT Image Processing

In the training process, the convergence change of the loss function can be obtained. With the increase of training times, the accuracy of the verification data obtained by the entire TJ-2 network was getting higher and higher. However, when the accuracy reached 80%, the accuracy can increase little. Until the end of the training, the loss function also gradually converged and showed a constant trend. The final accuracy was 82%. The training process of the TJ-2 full convolution network was completed. The learning changes of training the TJ-2 full convolution network indicated changes of three kinds of learning in TJ-2 network during training. The learning rate can control the loss function of the whole TJ-2 volume product neural network to decrease smoothly (Figure 4). The following image was about the aortic valve CT image and algorithm for CT image target region segmentation results. It revealed that the application of deep learning to calculate and process can clearly show the specific area of the lesion (Figure 5).

### 3.3. Measurement of Aortic Root Anatomy Using CT Images of Deep Learning Algorithm

The mean diameter calculated by the long and short diameter, the mean diameter calculated by the perimeter, and the mean diameter calculated by the area were used for paired test in CT. The results showed that the size of annulus in CT was larger, and there was no significant difference in the average diameter measured by three CT methods (23.2 ± 3.85, 24.12 ± 3.52, and 23.74 ± 2.25, *P* > 0.05) (Figure 6).

The diameter results calculated by the CT of the deep learning algorithm according to the measurement methods such as long-short diameter, area, and perimeter are shown in Table 2.

### 3.4. Complications

Among the 52 patients, there were 35 cases of hypertension, accounting for 67%, 13 cases of diabetes, accounting for 25%, 6 cases of chronic renal insufficiency (Cr > 2 mg/dL), accounting for 11% (including 2 cases of hemodialysis maintenance, accounting for 3.8%), 11 cases of chronic lung disease, accounting for 21%, 9 cases of cerebrovascular disease, accounting for 17.3%, and atrial flutter and atrial fibrillation. There were no patients with infective endocarditis (Table 3).

## 4. Discussion

At present, the preoperative screening of patients to undergo CT plays an important role, which can be used to provide important information for clinical sheath approach. It also provides anatomical information for the weight of ascending aorta, the size of aortic root, and aortic ring [14]. TAVI requires preoperative examination to assess the size of aortic rings noninvasively and accurately, which is of great significance for the size selection of TAVI valve rings. If the size of the valve ring is not good, it will cause complications around the ring, such as aortic regurgitation, valve embolism, and ring tearing. Computer tomography can provide accurate anatomical shape and size of aortic rings [15]. Previous studies suggested that the valve diameter selected by CT and two-dimensional ultrasound is larger than the ring diameter measured by ECG, which reduces aortic regurgitation [16]. Deep learning was widely used in medical fields, such as image or data processing, and achieved excellent processing results [17]. In this study, the TJ-2 full convolution network in deep learning was used to process CT images of patients. The results showed that the lesions in CT images can be effectively identified, which laid a foundation for subsequent research. Such results were consistent with the excellent results obtained by Guo et al. [18] who adopted the Elman neural network model in deep learning for image processing.

The repeatability of the diameter of the measured ring measured by the perimeter of scientific research evaluation is lower than that of the average diameter method and the area method. The average diameter measured by the area method is generally larger than that measured by the perimeter method in different cardiac cycles. In the contraction period, the elliptic index of the ring is minimal, which is closer to the circle than other cardiac cycles [19]. However, the diameter difference between the two calculated by the perimeter method and area method in the diastolic period is greater than that in the contraction period [20]. After stent implantation, especially after balloon implantation, the shape of the stent is round, and the same situation before and after surgery is the circumference of the ring. The ring diameter measured by the circle method may be more suitable for ring selection. The results of this study used the long-short diameter calculation, perimeter calculation, and area calculation in CT images to obtain the average diameter. The results represented that there was no significant difference in the average diameter measured by the three CT methods.

## 5. Conclusion

This study was to explore the use of deep learning in the measurement of information in CT images and its impact on surgical results. Of the 120 patients in this study, 52 eventually received TAVI treatment. The aortic ring diameter measured by three CT methods of deep learning algorithm is larger than that measured by CT, but there is no significant difference in the aortic ring diameter measured by their diameter measurement methods, and the area method and the long and short diameter method have high repeatability. Limitations are that although the size of the ring was chosen according to the different methods of measuring the ring, the most important thing is whether the final patient can undergo surgery, which is affected by many factors, including the vascular condition of the approach and the distortion angle of the blood vessel to the aorta, the diameter of the sinus orifice, and the width of the sinus orifice. This study summarizes and analyzes the characteristics of clinical complications and main influencing factors in patients with high-risk aortic valve stenosis and the preliminary experience according to moving root and anatomical data measurement. In the future, the sample size will be further expanded to integrate clinical data combined with intraoperative and clinical conditions, so that the preoperative evaluation results can better guide the screening of TAVI patients and standardize the success rate and prognosis of TAVI.

## Figures and Tables

**Figure 1:** TJ-2 fully convolutional network model.

**Figure 2:** Measurement process.

**Figure 3:** Results of three methods for measuring aortic valve ring.

**Figure 4:** Training TJ-2 full convolution network learning rate changes.

**Figure 5:** The CT images of aortic valves and the results of target region segmentation in CT images by the algorithm.

**Figure 6:** Average diameters measured by three CT methods.

**Table 1:** HEBIN basic data of patients.

Variable	Patient (*n* = 120)
Mean transvalvular pressure gradient (mm/hg)	57.65 ± 15.3
Gender (male)	67 (58%)
Height (cm)	164 ± 8.2
Body surface area (m^2^)	1.73 ± 0.15
Hypertension (%)	58 (48.3%)
Diabetes (%)	30 (25%)
Coronary heart disease (%)	32 (26.7%)
Peak velocity of aortic valve (m/s)	5.133 ± 0.65
Left ventricular ejection fraction (%)	54.3 ± 15.4

**Table 2:** Measurement of aortic root anatomy using CT images of the deep learning algorithm.

Measurement	95% CI (lower limit, upper limit)
Mean diameter calculated by the long and short diameter (mm)	0.88 (0.84, 0.92)
Mean diameter calculated by the perimeter (mm)	0.76 (0.68, 0.87)
Mean diameter calculated by the area (mm)	0.85 (0.72, 0.91)

**Table 3:** Complication information.

Item	Cases (*n* = 52)
Hypertension (%)	35 (67.3)
Diabetes (%)	13 (25.0)
Chronic renal insufficiency (Cr > 2 mg/dL) (%)	6 (11.5)
Hemodialysis maintenance (%)	2 (3.8)
Chronic lung disease (%)	11 (21.2)
Cerebrovascular disease (%)	9 (17.3)

## Data Availability

The data used to support the findings of this study are available from the corresponding author upon request.
